RETRACTED

# Cognition enhancing effects of *Clausena lansium* (Lour.) peel extract attenuate chronic restraint stress-induced memory deficit in rats

**DOI:** 10.1016/j.heliyon.2021.e07003

**Published:** 2021-05-11

**Authors:** W. Phachonpai, T. Tongun

**Affiliations:** a Division of Physiology, School of Medical Sciences, University of Phayao, Phayao, 56000, Thailand; b Department of Physiology, Faculty of Medicine, Khon Kaen University, Khon Kaen, 40002, Thailand

**Keywords:** *Clausena lansium* (Lour.) Skeel, Cognitive booster, Oxidative damage, Stress, Acetylcholinesterase inhibitors

## Abstract

Chronic stress exposure is now accepted as a problem that can produce deleterious effects on both brain structure and function. Numerous studies have proposed the potential of fruit peels as vital sources for acetylcholinesterase (AChE) inhibitors and antioxidants. *Clausena lansium* (Lour.) or wampee (WP) fruit peel is a rich source of antioxidants and flavonoids that could prove beneficial for human health. Currently, there has been no scientific evidence supporting the potency of WP peel extract to combat or reverse the memory impairment induced by chronic restraint stress (CRS). Therefore, we aimed to investigate the AChE-inhibiting and neuroprotective effects of WP peel extracts against CRS-mediated oxidative stress and cognitive dysfunction in rats. Initial assessment of the extract revealed antioxidant capacity and high concentrations of polyphenols. Further, Wistar rats were dosed orally with the WP peel extract (200, 400, and 600 mg/kg daily) and kept in a restrainer for 4 h a day for 28 consecutive days. The object recognition and Morris water maze tests were used to determine cognitive functions. After sacrifice, biomarkers of oxidative stress and AChE inhibitory activity in brain homogenates of rats were also investigated. CRS exposure produced oxidative stress and increased AChE activity, changes that led to learning and memory impairment in the cognition tests. Improved memory, reduced AChE activity, and a decreased oxidative stress status were seen in rats treated with WP peel extract. Overall, supplementation with WP peel extract may exert cognitive-enhancing effects through antioxidative neuroprotection and inhibition of AChE activity against CRS-induced oxidative stress.

## 1 Introduction

Exposure to chronic stress is a risk factor for the development of memory deficits (Azman et al., 2018). Chronic stress not only suppresses early long-term potentiation (LTP) (Pavlides et al., 2002), but it also reduces synaptic plasticity in the hippocampus (Wang et al., 2019). In addition, chronic stress exposure induces reactive oxygen species (ROS) overproduction and lowers brain antioxidant enzymes activities, alterations that have been associated with cognitive impairment (Wang et al., 2014).

RETRACTED

The neurotransmitter acetylcholine (ACh) plays an important role for the maintenance of accurate cognitive functions. *In vitro* and *in vivo* studies have shown that increased acetylcholinesterase (AChE) levels result in learning deficits and memory impairment (Croxson et al., 2011). Thus, acetylcholinesterase inhibitors (AChEIs) have been the mainstays of symptomatic therapy for cognitive disorders (Ashford, 2015).

In recent years, fruit peel waste from industries and household kitchen processes have gained attention as natural therapeutic agents that are rich in valuable bioactive components such as polyphenols, flavonoids, and vitamins, among many other compounds (Oliveira et al., 2009). These bioactive compounds have shown strong antioxidant activity (Parashar et al., 2014). In addition, several published studies have reported that various phytochemicals found in some fruit peels, including hawthorn, citrus, and banana, exhibit AChE-inhibiting activity (Wu et al., 2017). Therefore, the natural antioxidants and AChE-inhibiting components in fruit peels may be effective to protect or combat against the diseases, which are associated with oxidative stress.

*Clausena lansium* (Lour.) Skeels, also known as wampee (WP), belongs to the family Rutaceae; it is widely located in the northern Thailand and southern China. It is a well-known plant in Chinese and Thai traditional medicine for treating a variety of disorders, such as cough, asthma, malaria, hepatitis, and digestive problems (Jackobsen et al., 1972; Adebajo et al., 2009). It also exhibits several biological and pharmacological activities, including antitumour, antimicrobial, anti-inflammatory, hepatoprotective, antifungal, anti-obesity, neuroprotective, and antioxidant (Liu et al., 1996, 2019; Ng et al., 2003). WP peel extract has been shown to exert antioxidant and anticancer activities in *in vitro* models and in several cell lines: human gastric carcinoma (SGC-7901), human hepatoma (HepG2), and human lung adenocarcinoma (A549) (Prasad et al., 2009). However, there has been no scientific evidence to support cognitive-enhancing effects through WP fruit peel extract consumption. For the first time, this study explored the ability of WP peel extract to combat memory impairment induced by chronic restraint stress (CRS) through the inhibition of AChE activity or reduction of oxidative stress in rat brains.

## 2 Materials and methods

### 2.1 Drug and chemicals

Acetylthiocholine iodide (ATCI), bovine serum albumin (BSA), 5,5′-dithiobis (2-nitrobenzoic acid) (DTNB), 2,2-diphenyl-1-picrylhydrazyl (DPPH), the Folin–Ciocalteu reagent (FCR), thiobarbituric acid (TBA), 2,4-dinitrophenylhydrazine (DNPH), gallic acid, and vitamin C were purchased from Sigma-Aldrich (St. Louis, MO, USA).

RETRACTED

### 2.2 Preparation of the wampee fruit extract

Ripe WP fruit were harvested from a local farm in Amphoe Tanao, Nan Province, Thailand. WP peels were removed and washed carefully in running tap water and dried in a hot air oven at 40 °C. The dried samples were homogenized before maceration in a mixture of ethanol and distilled water for 48 h. The WP peel extract were filtered and concentrated using a rotary evaporator. The sample extract from the WP fruit peel produced a 10.93% yield; it was kept in a refrigerator at 4 °C in light-protected bottles for further study in the animals.

### 2.3 Total phenolic and flavonoid content determination

The total phenolic content was estimated using the Folin–Ciocalteu method (Lee et al., 2015), with some modification. Two-hundred microliters extract in water was mixed with 200 μL the Folin–Ciocalteu reagent. After 4 min, 2 mL Na_2_CO_3_ was added, and the mixture was incubated for 150 min in the dark at room temperature. The optical density was read at 765 nm and the results are expressed as mg gallic acid equivalents per 100 g dry weight (mg GAE/100 g DW).

The total flavonoid concentration of WP peel extract was measured with a colorimetric method (Shi et al., 2012), with slight modifications. In brief, 20 μL of the sample in 10 ml ethanol was mixed with 80 μL distilled water. Five microliters 15% (w/v) NaNO_2_ and 5 μL 10% (w/v) AlCI_3_ solutions were added to the mixture. After 5 min, 100 μL 4% (w/v) NaOH was added and adjusted the final volume to 200 μL. The mixture was incubated for 15 min and the absorbance was read at 510 nm using a spectrophotometer (Shimadzu Corporation, Kyoto, Japan). The total flavonoid content of the extracts is expressed as mg quercetin per 100 g DW (mg QE/100 g DW).

### 2.4 Determination of DPPH free radical scavenging activity

A modified DPPH assay (Öztürk et al., 2011) was used to assess the free radical scavenging ability of WP peel extracts. Five-hundred microliters of the extract was mixed with 500 μL DPPH (0.4 mM) in methanolic solution, vortexed, and incubated in the dark at room temperature for 30 min. The absorbance of the sample was read at 517 nm, and the percentage of scavenging activity of the extract was determined according to Eq. (1):

(1) $$\text{scavenging activity}\left(\text{\%}\right)=\left[\left({\text{A}}_{517\;\text{nm}}\;\text{of control}-{\text{A}}_{517\;\text{nm}}\;\text{of sample}\right)/{\text{A}}_{517\;\text{nm}}\;\text{of control}\right]\times 100$$

where A_517_ control is the absorbance of a control and A517 sample is the absorbance of WP peel extract sample.

RETRACTED

### 2.5 Experimental animals and protocol

All animal experiments were approved by the Institutional Animal Care and Use Committee of University of Phayao, and Khon kaen University, Thailand and were carried out in accordance with the principles of Laboratory Animal Care (National Institutes of Health publication, #85–23, revised in 1985).

A total of 48 male Wistar rats (7 weeks old, 220–250 g) were obtained from Nomura Siam International Co, Ltd. (Bangkok, Thailand). They were placed in standard metal cages (5 rats/cage) at an optimal temperature of 24 ± 2 °C, 45%–55% relative humidity, a 12-h light–dark cycle, and provided with commercial pellet diet and regular tap water.

After 1 week of acclimatizing to the new environmental conditions, the rats were randomly separated into six groups (n = 8 per group) as follows: (1) normal control unstressed group; (2) Vehicle (distilled water) + CRS (negative control); (3) Vit C (100 mg/kg) + CRS (positive control); (4) WP peel extract (200 mg/kg) + CRS; (5) WP peel extract (400 mg/kg) + CRS; and (6) WP peel extract (600 mg/kg) + CRS. The WP peel extract doses were effective based on our preliminary data. All rats received vehicle, positive control (Vit C), or WP peel extract via oral gavage once a day for 28 days. All substances were freshly prepared in a volume of 1 ml.

### 2.6 CRS induction

Approximately 30 min after oral administration of the appropriate treatment, rats of all the groups except the control group were subjected to CRS for 4 h per day (09:00 h to 13:00 h) for 28 consecutive days. Each rat was kept in the prone position in a well-ventilated Plexiglas tube (20 cm long, 7 cm in diameter) without access to food and water. After the restraint stress sessions, the rats were returned to their home cages with immediate access to water and food.

### 2.7 Determination of cognitive function

At the end of the study, the cognitive-enhancing effects of WP peel extract were evaluated by the object recognition test (ORT) and the Morris water maze (MWM) test. After cognition assessment, rats were sacrificed by decapitation and the whole brain was immediately removed to determine the AChE activity and oxidative stress status.

#### 2.7.1 ORT test

The ORT was performed in an open field arena box (50 × 50 × 50 cm) with a white floor. Two identical objects and one different object were used. Before the test, the rats were allowed to explore the empty arena for 5 min. In the familiarization trial, the rats were again allowed to explore the arena for 5 min, this time with two identical objects placed in separate locations. The object exploration time was judged when the rat sniffed or touched the object <2 cm from its nose. After 24 h, the rat was returned to the arena for 5 min; for this trial, one of the familiar objects was replaced with a novel object in the same location. The exploration time of each object was recorded using a stopwatch and presented as the discrimination index (DI). Eq. (2) used to calculate DI is:

(2) [(Time exploring the new object-Time exploring the familiar object)/Time exploring the novel object]

The ORT arena was cleaned with 10% ethanol to remove any remaining odours before each test.

RETRACTED

#### 2.7.2 MWM test

Spatial memory was tested using the MWM test (Morris, 1994). A circular metal tank (170 cm in diameter and 60 cm high) was filled with tap water (40 cm deep) and the surface of the water was covered with baby powder. The pool was separated into four quadrants. A removable platform was hidden 2 cm below the surface of the water level in a fixed location in one of the four quadrants. The rats must memorize the environmental cues to locate the platform. Each rat was placed in the water at one of the four quadrants and allowed to swim until it found the platform. The time for the rat to reach the underwater platform was regarded as the escape latency. Twenty-four hours later, the rats were tested to determine the retention memory. The platform was removed from the pool to determine spatial retention. The time spent in the target quadrant was recorded during a time period of 60 s. Cognitive impairment would be reflected by a longer escape latency and a shorter retention time.

### 2.8 Biochemical measurements

#### 2.8.1 Brain tissue preparation

After decapitation, the whole rat brain was immediately removed, washed with ice-cold 0.9% NaCl, weighed, and homogenized in ice-cold (4 °C) 50 mM sodium phosphate buffer (pH 7.4) with 0.2% Triton X-100 using a Potter–Elvehjem homogeniser. The brain homogenates were centrifuged at 9000 g for 30 min, and the supernatants were collected and stored at -70 °C to determine superoxide dismutase (SOD), catalase (CAT), glutathione peroxidase (GSH-Px), and AChE activities and the malondialdehyde (MDA) level.

#### 2.8.2 Lipid peroxidation determination

MDA, a marker of lipid peroxidation, was measured following the method of Okhawa et al. (1979). The reaction contained 0.2 mL brain homogenate, 0.2 ml ascorbic acid (100 mM), 0.2 mL 8.1% sodium dodecyl sulfate, and 0.58 ml phosphate buffer (0.1 M, pH 7.4). The mixture was shaken and incubated at room temperature for 60 min before adding 1.5 mL 0.8% thiobarbituric acid (TBA). The reaction was boiled in a water-bath for 30 min and then cooled with tap water before being centrifuged at 4000 g for 10 min. Absorbance was measured at 532 nm and the result is expressed as U/mg protein.

RETRACTED

#### 2.8.3 Antioxidant enzymes activities determination

SOD activity was determined following the method of Kakkar et al. (1984). Briefly, 10% brain tissue homogenate was mixed in 0.9% NaCl and then centrifuged at 15000 *g* for 15 min. The reaction mixture contained 1.2 ml sodium pyrophosphate buffer (0.052 mM, pH 7.0), 0.1 ml phenazine methosulphate (PMS, 186 μM), nitroblue tetrazolium (NBT, 300 μM), 0.5 ml brain homogenate, and 1.0 ml distilled water. It was incubated at room temperature for 5 min before adding 0.2 ml NADH (780 μM) to start the enzymatic reaction. After 2 min, 1.0 mL glacial acetic acid (17.4 M) was added to stop the reaction. The absorbance was read at 560 nm and the activity is expressed as U/mg protein.

CAT activity was determined according to the method of Aebi (1984) with slight modifications. Briefly, 0.1 mL 10% brain tissue homogenate was mixed in 1.15% KCl. The reaction contained 0.8 ml of 50 mM phosphate buffer (K_2_HPO^4^/NaH_2_PO_4_, pH 7.0) and 0.1 mL Triton X-100 (0.02%) and was incubated at room temperature for 10 min. The reaction was started by the addition of 0.4 ml H_2_O_2_ (5.9 mM). The absorbance of the reaction solution was recorded at 240 nm and the activity is expressed as U/mg protein.

GSH-Px activity was determined according to Paglia and Valentine (1967). The reaction comprised 0.3 ml phosphate buffer (0.1 M, pH 7.4), 0.05 ml sodium azide (2.25 M), 0.1 mL GSH (0,15M), 0.05 ml glutathione reductase (2 U/ml), 0.1 ml EDTA (1 mM), 0.1 mL NADPH (0.8 mM), 0.01 ml H_2_O_2_ (0.25 mM), and 0.05 mL brain homogenate. The mixture was vortexed and then incubated at room temperature for 10 min. The absorbance was read at 340 nm for 3 min and the activity is expressed as U/mg protein.

Protein in the brain tissues samples was estimated according to the method described by Lowry et al. (1951) using bovine serum albumin as a standard.

#### 2.8.4 AChE activity determination

AChE activity was determined based on the method of Ellman et al. (1961). The reaction contained 75 μL Tris-HCl (50 mM, pH 8), 25 μL ATCI (15 mM), 100 μL brain tissue homogenate, and 0.1% BSA in the wells of a 96-well plate. The plate was incubated at 25 °C for 5 min and the reaction was started after the addition of 0.03 mL DTNB and 0.05 mL ACTI. The absorbance was measured at 412 nm using spectrophotometer. The activity is expressed as U/mg protein.

### 2.9 Statistical analysis

Statistical evaluation was carried out using SPSS Statistics version 11 (SPSS Inc., Chicago, IL, USA). All data are expressed as mean ± standard error of the mean (SEM). The data were subjected to One-way analysis of variance (ANOVA) followed by post hoc analysis (Tukey's test). Differences were considered statistically significant at p < 0.05.

RETRACTED

## 3 Results

There were no adverse effects or deaths were observed in all of rats treated with various doses of WP peel extracts. These data suggest that the WP peel crude extract and the dosing schedule are safe.

### 3.1 The total phenolic and total flavonoid contents and antioxidant properties of WP peel extract

In the first part of this study, we evaluated the total phenolic content, the total flavonoid content, and the antioxidant activity of WP peel extract (Table 1). The WP peel extract had a strong ability to scavenge the DPPH radical (91.33% ± 0.27%). The WP peel extract contained a total phenolic content of 530.13 ± 0.07 mg GAE/100 g DW and a total flavonoid content of 49.73 ± 0.63 mg QE/100 g DW. It is very interesting that the peel of WP fruit is often discarded as waste even though it contains several beneficial phytochemical ingredients.

**Table 1:** Total phenolic compounds, total flavonoids, and antioxidant property of WP peel extracts.

Total phenolics (mg GAE/100 g DW)	Total flavonoids (mg QE/100 g DW)	DPPH (% scavenging activity)
530.13 ± 0.07	49.73 ± 0.63	91.33 ± 0.27

Values represent mean ± SD of three independent experiments.

### 3.2 Cognitive-enhancing effects of WP peel extract on spatial and non-spatial memory

The memory-enhancing effects of WP peel extract on non-spatial memory against CRS-induced memory deficits in rats is shown in Figure 1. The DI was significantly decreased (p < 0.05) in rats subjected to CRS and treated with vehicle compared with the control group, indicating that CRS exposure was associated with learning and memory impairment. However, the DI was significantly increased (p < 0.05) in rats subjected to CRS and treated with 100 mg/kg Vit C, serving as a positive control, and all doses of the WP peel extract compared with the rats subjected to CRS and treated with vehicle.

**Figure 1:** Effects of WP peel extract on the DI in the ORT in chronic restraint stressed rats. Values represent the mean ± SEM (n = 8). ^#^p < 0.05 vs control; ∗p < 0.05 vs vehicle + CRS group.

We also found a significant difference in spatial memory, evaluated with the MWM test, among the treated groups (Figure 2). Rats subjected to CRS and treated with vehicle showed a significantly longer escape latency compared with the control group (p < 0.05). In the retention trial, rats subjected to CRS and treated with vehicle showed a significantly shorter retention time compared with control group (p < 0.05). However, all doses of the WP peel extract ameliorated the cognitive dysfunction: the treated rats subjected to CRS showed a significantly shorter escape latency, but a longer retention time compared with the rats subjected to CRS and treated with vehicle (p < 0.05 all). There was a similar alteration in both escape latency and retention time in rats subjected to CRS and treated with Vit C (p < 0.05). These results indicate that CRS exposure severely impairs learning and memory and supplementation with WP peel extract attenuates these cognitive impairments.

RETRACTED

**Figure 2:** Effects of WP peel extract on the escape latency and retention time in the MWM test in chronic restraint stressed rats. Values represent the mean ± SEM (n = 8). ^#^p < 0.05 vs control; ∗p < 0.05 vs vehicle + CRS group.

### 3.3 The effects of WP peel extract on brain oxidation indices and antioxidant enzyme activities

Because oxidative stress is considered a major contributing factor to memory dysfunction, we also examined whether WP peel extract altered oxidative stress markers, including the level of MDA and the activities of SOD, CAT, and GSH-Px (Figure 3). The activity of the endogenous antioxidant enzymes in the brain of rats subjected to CRS and treated with vehicle were significantly reduced compared with the control group (p < 0.05). However, these activities were restored in the rats subjected to CRS and treated with WP peel extract compared with the rats subjected to CRS and treated with vehicle (p < 0.05 all). Similarly, the activities of SOD, CAT, and GSH-Px were elevated in the brain of rats subjected to CRS and treated with Vit C (p < 0.05).

**Figure 3:** Effects of WP peel extract on brain oxidative status in chronic restraint stress-treated rats. a) superoxide dismutase (SOD); b) catalase (CAT); c) glutathione peroxidase (GSH-Px); d) malondialdehyde (MDA). Values represent the mean ± SEM (n = 8). ^#^p < 0.05 vs control; ∗p < 0.05 vs vehicle + CRS group.

Depletion of antioxidant defenses leads to increased lipid peroxidation. We found that MDA levels in rats subjected to CRS and treated with vehicle were higher than those in control rats (p < 0.05). Again, rats subjected to CRS and treated with Vit C or WP peel extract (all doses) showed a significantly reduced MDA level in the brain (p < 0.05 all) compared with rats subjected to CRS and treated with vehicle.

### 3.4 Anti-AChE activity of WP peel extract

The WP peel extract was also assessed for its potential to inhibit AChE, an enzyme related to cognitive impairment. Rats subjected to CRS and treated with vehicle exhibited high AChE activity in the brain compared with the control group (p < 0.05). Surprisingly, all WP peel extract doses significantly (p < 0.05) inhibited AChE activity in rats subjected to CRS compared with rats subjected to CRS and treated with vehicle (Figure 4).

RETRACTED

**Figure 4:** Effects of WP peel extract on brain AChE activity in chronic restraint stressed rats. Values represent the mean ± SEM (n = 8). ^#^p < 0.05 vs control; ∗p < 0.05 vs vehicle + CRS group.

## 4 Discussion

A myriad of studies has revealed that fruit peel waste is a good source of bioactive compounds with antioxidant activity that may help in preventing various diseases (Larrosa et al., 2002; Al-Sayed and Ahmed, 2013). The results of this study revealed that WP peel extract is a candidate functional food product to improve memory distortion caused by exposure to CRS.

Numerous studies have shown that there is a strong relationship between antioxidant activities and phenolic and flavonoid contents in fruit and vegetable wastes (Ain et al., 2020; Azizan et al., 2020). The antioxidant capacity of WP peel extracts in this study is in agreement with the total phenolic and flavonoid contents reported in Table 1. Our results are also consistent with the study by Prasad et al. (2009b), who reported that the total phenolic content of a butanol extract of WP peel was 30.3 ± 5.4 μg/g DW and the DPPH scavenging activity was 95% ± 0.65%. The differences compared with our results are probably due to different extraction methods, standard solutions, climate conditions, and geographical variation in plant species.

It has been widely accepted that long-term stress exposure stimulates excessive production of free radicals, a phenomenon that leads to cognitive dysfunction (Moench et al., 2019). CRS is a classic and simple method that can induce learning and memory impairment (Wang et al., 2014) through several mechanisms, for example, the activation of the hypothalamic–pituitary–adrenal (HPA) axis and increased free radical production, leading to oxidative stress in the brain (Seckl et al., 1993). Our results showed that exposure to CRS is linked to memory decline in both non-spatial and spatial memory. After 4 weeks of CRS exposure, the rats in the vehicle-treated group showed more amnesic behavior, denoted by a decreased DI in the ORT and an increased escape latency but reduced retention time in MWM test. These cognitive behavioral changes were paralleled by biochemical alterations, including a higher level of MDA (a brain lipid peroxidation marker) accompanied by lower SOD, CAT, and GSH-Px activities. Our data are consistent with previous studies (Liang et al., 2015). In addition, these results suggest that the CRS paradigm is suitable to determine the cognition-enhancing effects of WP peel extract against CRS-induced memory impairment in rats.

RETRACTED

There is increasing scientific attention to developing food supplementation based on fruit and vegetable wastes, which exert antioxidant effects (Cheok et al., 2018; Saini et al., 2019). The present report shows that WP peel extract possesses strong antioxidant abilities and a relatively high margin of safety. The WP peel extract ameliorated the cognitive behavioral and biochemical alterations in the rats subjected to CRS. All doses of the WP peel extract significantly increased the DI in the ORT. In addition, various doses of this extract significantly reduced the escape latency and increased the retention time in the MWM test. The decreased MDA level as well as increased endogenous antioxidant enzyme activities confirmed the WP peel extract–mediated neuroprotective effect in the rats subjected to the CRS paradigm.

ACh is a crucial neurotransmitter in cognition (Schliebs and Arendt, 2011); thus, the idea of increasing the ACh concentration in the brain to restore memory impairment has gained tremendous interest. This has led to the development of drugs or substances able to inhibit or decrease AChE activity to maintain ACh levels. In this study, AChE activity was elevated in the brain of rats subjected to CRS and treated with vehicle. The decreased AChE activity in the brain of rats subjected to CRS and treated with WP peel extract (all doses) is likely a response related to a decrease in ROS production due to elevated endogenous antioxidant enzyme activities.

Taken together, our findings demonstrate that the oral supplementation with WP peel extract at various doses (200, 400, and 600 mg/kg BW) attenuates CRS-induced cognitive impairment, as indicated by restored memory function in spatial and non-spatial learning and memory tests. We also established that the mechanisms by which the WP extract enhances cognition may be mediated by reducing brain oxidative stress and increasing brain antioxidant status, along with anti-AChE activity.

While the highest dose of WP peel extract (600 mg/kg BW) showed greater efficacy in all parameters, there was not a dose-dependent effect. This finding suggests that the crude extract of WP peel used in this experiment contains numerous important bioactive constituents. Some of these constituents are inactive, but some of them are active, depending on the relationship between functional groups and the target binding site of the active compounds. Thus, the antioxidant and the cognitive-enhancing effects of WP peel extract may occur via additive, synergistic, or antagonistic interactions among different bioactive compounds of the crude extract; these interactions, in turn, alter the neurophysiological effects. While we had aimed to identify the active constituents of the WP peel extract, the COVID-19 pandemic and the infection control policy of our laboratory unit has unfortunately limited our study. Therefore, there is a further need to identify the active compounds from WP peel extract that are responsible for a given cognitive-enhancing effects. Moreover, further studies are required to investigate the effects by which WP peel extract could regulate the HPA axis in a rat model of CRS.

RETRACTED

## 5 Conclusion

Overall, the results of our study indicate that crude WP peel extract contains polyphenolic compounds that exhibit strong antioxidant capacities and anti-AChE activity, which can be developed in nutraceutical products to enhance cognition. Thus, it is time to devote more effort towards understanding the mechanisms of action of the bioactive compounds that are present in this extracts.

## Declarations

### Author contribution statement

W. Phachonpaia: Conceived and designed the experiments; Performed the experiments; Analyzed and interpreted the data; Contributed reagents, materials, analysis tools or data; Wrote the paper.

T. Tong-unb: Performed the experiments; Analyzed and interpreted the data; Contributed reagents, materials, analysis tools or data.

### Funding statement

This research did not receive any specific grant from funding agencies in the public, commercial, or not-for-profit sectors.

### Data availability statement

The authors do not have permission to share data.

### Declaration of interests statement

The authors declare no conflict of interest.

### Additional information

No additional information is available for this paper.
